# Esthetic Root Coverage with Double Papillary Subepithelial Connective Tissue Graft: A Case Report

**DOI:** 10.1155/2014/509319

**Published:** 2014-02-04

**Authors:** Ramesh Babu Mutthineni, Ram Babu Dudala, Arpita Ramisetty

**Affiliations:** ^1^Department of Periodontics, Mamata Dental College, Khammam, Andhra Pradesh 507002, India; ^2^Department of Periodontics, Haldia Institute of Dental Sciences, Purba Medinipur, West Bengal 721645, India; ^3^Mamata Dental College, Khammam, Andhra Pradesh 507002, India

## Abstract

Patients today have become excessively concerned about esthetics. These esthetic concerns of patients have become an integral part of periodontal practice. Gingival recession is an esthetic problem that can be successfully treated by means of several mucogingival surgical approaches, any of which can be used, provided that the biologic conditions for accomplishing root coverage are satisfied with no loss of soft and hard tissue height interdentally. There are currently different techniques for root coverage which include pedicle grafts, free gingival grafts, connective tissue grafts, and guided tissue regeneration (GTR). This paper reports a case in which a new double papillary connective tissue graft technique has been used in the treatment of gingival recession.

## 1. Introduction

The principal aim in surgically treating gingival recession is to cover the exposed root surfaces and consequently improve esthetic appearance, although there are other objectives such as inhibiting the progression of active recession, increasing the width of attached gingiva, and reducing dental hypersensitivity. Several techniques such as free gingival graft [1–3], laterally positioned flap [4–6], coronally positioned flap [7, 8], and double papilla graft [9] have been proposed for the same.

The objective of free gingival graft procedure is to prevent future recession by increasing the width of keratinized gingiva rather than covering the root surface. A double-step procedure consisting of a free gingival graft to obtain a sufficient amount of keratinized tissue, if not already present, and a coronally positioned flap performed after healing to cover the exposed root surface has been proposed. Many variations of the grafting technique have been proposed for predictable root coverage [10–12]. In 1985, B. Langer and L. Langer [13] presented a surgical combination of a pedicle flap and a free graft, proposing that subepithelial connective tissue graft covering the lesion is overlapped by a partial thickness flap to ensure vascularization of the free graft. Different flap procedures further modified this technique resulting in a high success rate and predictability as shown in various longitudinal observations and case reports [14–17].

Recently, double papillary connective tissue graft has been used for the treatment of root coverage procedures for better esthetics and predictability. Of the various graft and nongraft procedures used, this case report describes double papillary subepithelial connective tissue graft, a technique in which bilateral pedicle flaps with connective tissue graft were used to cover Miller's class II gingival recession in the lower left lateral incisor.

## 2. Case Report

A-25-year old male patient reported to the Department of Periodontics, Mamata Dental College and Hospital, Khammam, Andhra Pradesh, with the chief complaint of receding gum and hypersensitivity in relation to lower left lateral incisor (tooth number 32). The patient was a nonsmoker with a good general health and had received no antibiotics and/or periodontal therapy during the previous six months. On intraoral examination, Miller's class II recession was seen in relation to tooth number 32. Trauma from occlusion and tooth malposition with respect to the involved tooth was ruled out clinically. Prior to therapy, clinical measurements including probing depth (2 mm), recession depth (5 mm), recession width (3 mm), clinical attachment level (CAL, 7 mm), and width of keratinized tissue (3 mm) were obtained using a Williams periodontal probe. Clinical photographs were taken preoperatively (Figure 1) and postoperatively (Figure 10). Intraoral periapical radiograph (IOPA) of the area showed no bone loss in relation to number 32 (Figure 2).

### 2.1. Presurgical Preparation

The patient was educated and motivated about the procedure and informed consent was obtained. Oral hygiene instructions with emphasis to brushing habits were given. Thorough scaling and root planing were done. The patient was periodically recalled to assess the oral hygiene and gingival status.

### 2.2. Surgical Technique

The proposed flap design for the surgical procedure has been shown in Figure 3. Following local anesthesia, an intracrevicular incision through the bottom of the crevice followed by mesial and distal vertical releasing incisions were made including both papillae adjacent to 32 (Figure 4). A partial thickness flap was reflected by sharp dissection as close to the periosteum as possible, beyond the mucogingival junction, and was extended until the partial thickness flap could be passively positioned over the defect without tension (Figure 5). Following flap elevation, the exposed root surface was gently planed with sharp curettes. The exposed root surface was then conditioned with 50 mg/mL tetracycline solution for 3 minutes with subsequent saline rinsing using a three-way syringe.

Subepithelial connective tissue graft was obtained (Figure 7) in the region of number 24 and number 25 from the palate with two incisions (L-shape) (Figure 6), to prevent severe postoperative pain and discomfort and for early wound healing. The harvested connective tissue graft was sutured over the defect using a 5-0 vicryl suture to cover the graft, both papillae were first sutured midbuccally in relation to number 32 (Figure 8) followed by suturing of vertical incisions using 5-0 mersilk suture without tension (Figure 9). A periodontal dressing (Coe-Pak) was applied to the surgical site to protect the site from irritation.

Patient was instructed to discontinue tooth brushing and to avoid trauma or pressure at the surgical site. A 0.12% chlorhexidine rinse was prescribed twice daily for 2 weeks and amoxicillin 500 mg thrice daily for 5 days to prevent infection. The patient was recalled after 10 days for suture removal. The patient was enrolled in a maintenance programme (professional plaque control and oral hygiene instructions) and was instructed to resume mechanical tooth cleansing with a soft toothbrush using the roll technique after 2 weeks.

## 3. Discussion

Indications for periodontal esthetic surgery for recession coverage include small amount of keratinized gingiva, class I or class II gingival recession, esthetic concern, single or multiple recessions, and root hypersensitivity. The contraindications include smoking and desquamative gingivitis [18–20]. The associated etiologic factors for gingival recession are faulty tooth brushing, malpositioning of tooth, friction from soft tissue, gingival inflammation, high frenum attachment, trauma from occlusion, and orthodontic tooth movement [21, 22]. The prevalence of gingival recession is more common among girls and the prevalence is seen to increase with age [23].

The rationale behind using a subepithelial connective tissue graft for recession coverage is that this technique combines the free gingival graft and pedicle flap. Regardless of the amount of attached gingiva present, the free autogenous connective tissue is readily available from palate or edentulous ridge and pedicle available from site is immediately apical to the gingival recession.

The vitality and high survival potential of subepithelial connective tissue graft are achieved by the double sources of the blood supply from the gingival flap facially and the overlying periosteum on the opposite side. Another advantage of this procedure is the maintenance of gingival esthetics during the healing process, thus avoiding the keloid appearance of the grafted tissue. Although subepithelial connective tissue grafts provide excellent esthetics, the amount of donor material necessary limits the number of teeth that can be treated in a single surgery.

The double papilla flap procedure was first described by Tackas 1995 [24]. It was designed to achieve an adequate zone of attached keratinized gingiva and/or coverage of a denuded root surface by joining two interdental papillae. Indications for this procedure include (1) when the interproximal papillae adjacent to the mucogingival problem are sufficiently wide, (2) when the attached gingiva on an approximating tooth is insufficient to allow for a laterally positioned flap, and (3) when periodontal pockets are not present.

The surgical procedure in the present study was performed according to the technique described by Tackas (1995) using connective tissue graft covered by a double pedicle papilla flap [24]. At the end of 6 months, the recession was completely covered and the width of keratinized gingiva increased by 4 mm (Figure 10). The advantages seen with this technique are little alveolar bone loss due to minimal exposure of the underlying periosteum, high predictability, greater availability of attached gingiva, and rapid wound healing at the donor site. The primary disadvantage with this technique is the technical expertise required in joining together two small flaps in such a way that they acted as a single flap [9].

## 4. Conclusion

The present case report demonstrated that the double papillary flap in conjunction with subepithelial connective tissue graft is an effective treatment modality for the management of recession defects affecting teeth in the esthetic zones of the mouth. In fact, this surgical technique resulted in complete root coverage of the treated case.

## Figures and Tables

**Figure 1:** Preoperative photograph showing recession in relation to 32.

**Figure 2:** Radiograph in relation to lower anterior region showing absence of interdental bone loss.

**Figure 3:** Proposed flap design for double papillary in relation to tooth number 32.

**Figure 4:** Intracrevicular incision followed by mesial and distal vertical releasing incisions for double papilla flap in relation to tooth number 32.

**Figure 5:** Partial thickness flap reflection in relation to tooth number 32.

**Figure 6:** Donor site in the palate used for harvesting the subepithelial connective tissue graft.

**Figure 7:** Harvested free connective tissue graft.

**Figure 8:** Papillary grafts from adjacent papillae first sutured midbuccally in relation to recipient site.

**Figure 9:** Suturing of vertical incisions using 5-0 mersilk suture without tension.

**Figure 10:** Sixth month postoperative view showing complete recession coverage in relation to tooth number 32.
